The article "Analysis of Risk Factors and Protective Strategies for Tube Blockage in Patients with Drug-Induced Liver Failure Based on Artificial Liver Therapy" was retracted in 2023. Reasons: signs of a paper mill; compromised peer review; unreliable results or conclusions.

# Analysis of Risk Factors and Protective Strategies for Tube Blockage in Patients with Drug-Induced Liver Failure Based on Artificial Liver Therapy

**DOI:** 10.1155/2023/8201776

**Published:** 2023-04-08

**Authors:** Yan Shen, Liping Shi, Luxi Deng, Xiaoling Zhao

**Affiliations:** Department of Infectious Diseases, The First Affiliated Hospital of Nanjing Medical University, Nanjing 210029, Jiangsu, China

## Abstract

**Objective:**

To analyse the influencing factors of tube blockage during the treatment of artificial liver in patients with drug-induced liver failure and explore effective patient protection strategies.

**Methods:**

In this study, 49 patients with pharmacological (antituberculosis drugs, antibiotics, proprietary Chinese medicine, gastric drugs, and antihyperthyroid drugs) liver failure admitted to our hospital from June 2015 to December 2021 were selected for prospective analysis. Clinical indicators and general data of all patients were collected and collated, risk factors leading to the obstruction of artificial liver treatment were analysed, and corresponding protective measures were proposed.

**Results:**

The incidence of tube blockage was 5.32% (10 times) in 49 patients with pharmacological liver failure treated 188 times with artificial liver therapy. The incidence of tube blockage was significantly higher in patients in the PDF mode than in those in the PP and PE modes (*P* < 0.05), and there were differences in the location of blocked tubes between the treatment modes. Blocked tubes occurred more often in the venous cauldron of the circuit in the PDF mode and in the plasma separator of the circuit in the PP mode. The incidence of tube blockage was significantly lower in patients with no more than 3 treatments than in those with 3 to 5 treatments and those with more than 5 treatments (*p* < 0.05). The incidence of catheter blockage was higher in patients with PTA values ≤20% than in those with PTA values between 20% and 30%, and higher than in those with PTA values above 30% (*P* < 0.05).

**Conclusion:**

The risk factors of tube plugging in patients with liver failure treated with artificial liver include different treatment modes, different treatment times, and different PTA values. The PDF mode has a higher rate of tube plugging than PE or PP treatment modes. The more the number of treatment times and the lower the PTA value of patients, the more tube plugging is likely to occur.

## 1. Introduction

The liver is the primary organ of drug metabolism and is therefore highly susceptible to damage by the drug itself or its metabolites, predisposing it to liver failure based on chronic liver disease [1]. Liver failure is a life-threatening clinical syndrome caused by severe impairment or failure to compensate for important liver functions such as biosynthesis, specific detoxification, excretion, and filtration, and may be triggered by a variety of factors such as viral infections, alcohol, drugs, and hepatotoxic substances [2]. Liver failure is rapidly progressive and difficult to treat, and the overall prognosis for patients is poor [3]. In China, acute (subacute) liver failure and chronic liver failure are predominantly in males, and the age of onset is predominantly in young and middle-aged [4]people. There are no reliable prognostic indicators or systems for assessing liver failure, but overall, it is a group of diseases with a poor prognosis [5].

The article "Analysis of Risk Factors and Protective Strategies for Tube Blockage in Patients with Drug-Induced Liver Failure Based on Artificial Liver Therapy" was retracted in 2023. Reasons: signs of a paper mill; compromised peer review; unreliable results or conclusions.

In recent years, artificial livers have been widely used in the treatment of patients with drug-related liver failure and have become the standard of care for the treatment of acute liver failure [3]. The common treatment modalities for the artificial liver are plasma permeation (PDF), plasma perfusion (PP), and plasma exchange/selective plasma exchange (PE) [6–8]. The PE mode of treatment involves drawing the patient's blood, separating the plasma and cellular components with a plasma separator, discarding the patient's plasma, and then injecting fresh plasma into the patient to reduce pathological damage and eliminate pathogenic substances [9]. The PP mode treatment involves the separation of plasma from whole blood followed by adsorption of various toxins from the plasma through a perfusion device; the plasma will then fuse with the tangible fractions of the blood and return to the patient [10]. The PDF mode involves filtering some of the plasma containing protein-bound toxins out of the membrane and discarding it, removing the water-soluble toxins to varying degrees by diffusion and convection, and replenishing the replacement fluid (fresh frozen plasma, albumin fluid, etc.) into the patient [11]. However, there are certain risks associated with artificial liver therapy, such as catheter blockage, allergic reactions, swelling at the puncture site, bleeding, pulmonary hemorrhage, and secondary infection, which seriously affect the patient's treatment outcome and prognosis. In view of this, this paper analyses the risk factors for catheter occlusion in patients undergoing artificial liver therapy for drug-related liver failure and proposes targeted protection strategies.

## 2. Materials and Methods

### 2.1. General Information

In this study, 206 patients with liver failure admitted to our hospital from June 2015 to December 2021 were selected for prospective analysis, of which 49 cases were diagnosed as drug-related liver failure. There were 30 male patients and 19 female patients, ranging in age from 8 to 87 years old, with an average age of 47.52 ± 2.67 years.

49 patients had a clear medication history before treatment, mainly including (1) antituberculosis drugs (mainly isoniazid and rifampin, a total of 31 cases); (2) antibiotics (mainly erythromycin, doxorubicin, and itraconazole, a total of 7 cases); (3) 5 cases of Chinese patent medicines; (4) 4 cases of gastric disease drugs; and (5) 2 cases of thiourea antihyperthyroidism drugs. The study was approved by the Ethics Committee of the First Affiliated Hospital of Nanjing Medical University, No. 8791991.

The article "Analysis of Risk Factors and Protective Strategies for Tube Blockage in Patients with Drug-Induced Liver Failure Based on Artificial Liver Therapy" was retracted in 2023. Reasons: signs of a paper mill; compromised peer review; unreliable results or conclusions.

### 2.2. Methods

All patients were treated with comprehensive medical treatment. At the same time, the best combination of artificial liver support therapy was determined according to the actual progress of the patient's condition. A total of 188 artificial liver treatments were performed, including 61 times PE (plasma exchange) treatment, 52 times PDF (plasma diafiltration) treatment, and 75 times PP (plasma bilirubin adsorption) treatment.

The prothrombin time (PT) of all patients was detected, and the PTA value of prothrombin activity was calculated.

The instruments selected in this study included the Plasauto iQ21 blood purification machine (Asahi Kasei Medical, Tokyo, Japan).

### 2.3. Statistical Analysis

All data were analysed using SPSS 20.0. Enumerated data were expressed as numbers/percentages (*n*/%). Comparisons were made using the chi-squared test. Normally distributed measurements were calculated as mean ± standard deviation ($\bar{x}$ ± *s*). Comparisons between the groups were made using independent samples *t*-tests, and comparisons before and after the same group were made using paired *t*-tests. Differences were considered statistically significant when *P* < 0.05.

## 3. Results

### 3.1. General Data

A total of 49 patients with liver failure received artificial liver therapy 188 times; 10 times tube blockage occurred, and the incidence of tube blockage was 5.32%. Nineteen patients received no more than 3 treatments, 26 received 3–5 treatments, and 4 received more than 5 treatments (Table 1).

### 3.2. Comparison of the Incidence of Tube Blockage under Different Treatment Modes

The incidence of pipe blockage was 9.62% (5/52) in the PDF mode, 4% (3/75) in the PP mode, and 3.28% (2/61) in the PE mode. The PDF model is statistically more at risk of pipe blockage compared to the PE and PP modes (*P* < 0.05). Moreover, in the PDF mode, tube plugging mostly occurs in the venous kettle of the circuit, and in the PP mode, tube plugging mostly occurs in the plasma separator of the circuit (Table 2).

The article "Analysis of Risk Factors and Protective Strategies for Tube Blockage in Patients with Drug-Induced Liver Failure Based on Artificial Liver Therapy" was retracted in 2023. Reasons: signs of a paper mill; compromised peer review; unreliable results or conclusions.

### 3.3. Comparison of the Incidence of Tube Blockage under Different Treatment Times

The incidence of blockage in patients with no more than 3 treatments was 2.04%, which was lower than the incidence of blockage in patients with 3–5 treatments (4.49%) and significantly lower than the incidence of blockage in patients with more than 5 treatments (16%) (*P* < 0.05) (Table 3).

### 3.4. Comparison of the Incidence of Blocked Pipes under Different PTA Values

The incidence of tube blockage in patients with the PTA value no more than 20% was 7.81% (5/64), which was higher than 5.48% (4/73) in patients with the PTA value ranging from 20% to 30% and higher than 1.96% (1/51) in patients with the PTA value higher than 30% (*P* < 0.05) (Table 4).

## 4. Discussion

There is no specific treatment for liver failure, but in principle, early diagnosis and treatment are important, with appropriate etiological and comprehensive treatment measures to delay the exacerbation of the disease and actively prevent and treat complications [12]. The prognosis of liver failure depends on a “contest” between the degree of hepatocyte necrosis and the ability to regenerate, with a gradual recovery if hepatocyte regeneration exceeds necrosis and a poor prognosis if the disease deteriorates [13]. A common treatment option for liver failure is artificial liver plasma exchange, and artificial liver therapy is becoming more common in drug-related liver failure [3]. Artificial liver therapy is widely used in clinical practice as it can increase the overall efficiency of treatment and help improve patient prognosis [14]. However, artificial liver therapy requires puncture, which is an invasive procedure and therefore has a complex impact on the treatment outcome [15]. Patients are highly susceptible to blockage, allergic reactions, haematoma at the puncture site, and decreased blood pressure [16]. Blockage is the most common and adequate protective measures must be taken to prevent catheter blockage from affecting patient outcomes.

In this study, 49 patients with drug-related liver failure received 188 treatments with artificial liver, and the incidence of tubular occlusion was 5.32% (10). The main risk factors included the mode of treatment, number of treatments, and PTA values (prothrombin activity). The incidence of tube blockage was 9.62% (5/52) in the PDF mode, which was significantly higher than 4.00% (3/75) in the PP mode and 3.28% (2/61) in the PE mode (*P* < 0.05), with differences in the location of blocked tubes between treatment modalities. Blocked tubes occurred more often in the venous cauldron of the circuit in the PDF mode and in the plasma separator of the circuit in the PP mode. The incidence of blocked tubes was 2.04% (1/49) in patients with no more than 3 treatments, which was significantly lower than 4.39% (5/115) in patients with 3 to 5 treatments and 16% (4/25) in patients with more than 16 treatments. The incidence of catheter occlusion was 7.81% (5/64) in patients with PTA values ≤20%, which was higher than 5.48% (4/73) in patients with PTA values between 20% and 30%, and higher than 1.96% (1/51) in patients with PTA values above 30% (*P* < 0.05). In other words, the more the number of treatments in the PDF treatment modality, the lower the PTA values of the patients and the more likely they were to develop catheter occlusion.

The article "Analysis of Risk Factors and Protective Strategies for Tube Blockage in Patients with Drug-Induced Liver Failure Based on Artificial Liver Therapy" was retracted in 2023. Reasons: signs of a paper mill; compromised peer review; unreliable results or conclusions.

The protective measures to avoid the above situations are as follows: first, when the intubation time is long and the blood source is relatively tight, the clinician should confirm with the blood transfusion department before treatment that there is no problem with the blood supply before starting the intubation. Before catheterization, the nurse in charge needs to confirm whether the patient's coagulation mechanism and platelet count are normal [17]. Second, strengthen the training of pretreatment personnel to strictly abide by the technical specifications of artificial liver surgery, formulate alarm treatment and complication treatment plans for mechanical equipment, and establish appropriate artificial hepatic vascular access to ensure adequate drainage; extracorporeal circulation pipelines must be installed correctly. Make sure that the tubing is heparinized and that no air is present after the tubing is flushed [15]. On the other hand, during the treatment, the patient should be re-evaluated and given ECG monitoring, closely monitor the changes of the patient's vital signs, observe whether the patient has adverse reactions, and monitor various pressures (including transmembrane pressure and arterial pressure, venous pressure, secondary membrane inlet pressure) changes, deal with various alarms in time, reduce the number of pump stops, and shorten the treatment time [18]. Finally, after treatment, keep the artificial liver indwelling catheter properly. Catheter care was performed in accordance with the ISO9001 Nursing Quality Management System [19]. Pay attention to observe the fixation of the indwelling catheter, whether there is loosening or falling off, etc., inform the patient and family members of the precautions, and use a restraint strap to assist in the fixation if necessary; properly massage and guide the patient to perform active and passive functional exercises of the limbs to ensure adequate blood circulation and to reduce the risk of thrombosis; catheter patency checks and care are performed every other day [20].

The article "Analysis of Risk Factors and Protective Strategies for Tube Blockage in Patients with Drug-Induced Liver Failure Based on Artificial Liver Therapy" was retracted in 2023. Reasons: signs of a paper mill; compromised peer review; unreliable results or conclusions.

According to TCM, the main causes of liver failure are heat, toxicity, blood stasis, and phlegm, so accordingly, detoxification, elimination of blood stasis, and dispelling phlegm are the main rules of treatment for liver failure [21]. In the treatment of complications caused by liver failure, such as upper gastrointestinal bleeding and hepatic encephalopathy, while clearing heat, reducing yellowing, detoxifying toxins, and resolving stasis, it is necessary to stop bleeding, open the internal organs, and open the orifices at the same time [22]. After liver failure has occurred, there are several TCM treatments that can be taken, including the following: patients can be treated with acupuncture or moxibustion, which can be helpful in treating liver failure [23]; if patients experience significant abdominal distention, they can be treated with an enema using Chinese herbs, which can promote the recovery of gastrointestinal function, reduce abdominal distention, and alleviate intraabdominal pressure [24]; patients can also be treated with oral Chinese medicine, but there needs to be a principle that mainly takes the form of clearing heat, relieving dampness, reducing yellowing, and resolving blood stasis, and it needs to be dialectically substantiated so that good results can be achieved [25]. In addition, TCM is only an adjunctive treatment. After liver failure has occurred, the most important treatment is Western medicine.

However, there are some limitations to our study. First, our sample size was small, leading to a greater degree of chance in the experiment. Second. we should have considered more influential factors, including regional and age differences, and based on this we will establish more detailed inclusion criteria for all subsequent experiments. Finally, we also need to conduct a large number of follow-ups to determine the accuracy of the results.

## 5. Conclusion

In summary, risk factors were evaluated for catheter blockage in patients with liver failure treated with artificial liver include different treatment modalities, different treatment times, differences in PTA values, and a higher rate of blockage in the PDF compared to the PE or PP treatments modes, while the more number of treatments the lower the patient's PTA value, the more likely they are to experience tube blockage.

## Figures and Tables

**Table 1:** General information.

	Patients with drug-inducedliver failure (*N* = 49)
Gender	
Male	30
Female	19
Average age	47.52 (±2.67)
Drug history	
Antituberculosis drugs	31
Isoniazid	13
Rifampin	10
Antibiotic drug	7
Erythromycin and adriamycin	4
Itraconazole	2
Proprietary Chinese medicine	5
Stomach medicine	4
Thiourea antihyperthyroid drugs	2
Manual treatment method (times)	
PE	61
PDF	52
PP	75

The article "Analysis of Risk Factors and Protective Strategies for Tube Blockage in Patients with Drug-Induced Liver Failure Based on Artificial Liver Therapy" was retracted in 2023. Reasons: signs of a paper mill; compromised peer review; unreliable results or conclusions.

**Table 2:** Occurrence of tube blockage under different treatment modes.

Treatment modes	Number ofblocked pipes	Total numberof treatments
PE	2	61
PDF	5	52
PP	3	75
*P* value	*P* < 0.05	
*x* ^2^		

**Table 3:** Occurrence of tube blockage under different treatment times.

Treatment times	Number of blocked pipes	Total numberof treatments
≤3 times	1	49
>3 and ≤5 times	5	114
>5 times	4	25
*P* value	*P* < 0.05	
*x* ^2^		

**Table 4:** Occurrence of blocked pipes under different PTA values.

Prothrombin activity PTA value	Number of blocked pipes	Total number of treatments
PTA ≤ 20%	5	64
20% ≤ PTA ≤ 30%	4	73
PTA > 30%	1	51
*P* value	*P* < 0.05	
*t*		

## Data Availability

All data generated or analysed during this study are included in this published article.
